# MSIS: Multispectral Instance Segmentation Method for Power Equipment

**DOI:** 10.1155/2022/2864717

**Published:** 2022-01-04

**Authors:** Jun Shu, Juncheng He, Ling Li

**Affiliations:** ^1^School of Electrical and Electronic Engineering, Hubei University of Technology, Wuhan 430068, China; ^2^Hubei Key Laboratory for High-efficiency Utilization of Solar Energy and Operation Control of Energy Storage System, Hubei University of Technology, Wuhan 430068, China

## Abstract

Infrared image of power equipment is widely used in power equipment fault detection, and segmentation of infrared images is an important step in power equipment thermal fault detection. Nevertheless, since the overlap of the equipment, the complex background, and the low contrast of the infrared image, the current method still cannot complete the detection and segmentation of the power equipment well. To better segment the power equipment in the infrared image, in this paper, a multispectral instance segmentation (MSIS) based on SOLOv2 is designed, which is an end-to-end and single-stage network. First, we provide a novel structure of multispectral feature extraction, which can simultaneously obtain rich features in visible images and infrared images. Secondly, a module of feature fusion (MARFN) has been constructed to fully obtain fusion features. Finally, the combination of multispectral feature extraction, the module of feature fusion (MARFN), and instance segmentation (SOLOv2) realize multispectral instance segmentation of power equipment. The experimental results show that the proposed MSIS model has an excellent performance in the instance segmentation of power equipment. The MSIS based on ResNet-50 has 40.06% AP.

## 1. Introduction

In the fault detection of power systems, infrared imaging technology has the characteristics of operationally simple, fast response speed, and accurate judgment; it has become an important tool for the systems of failure detection [1]. By processing the collected images, the fault status of the power equipment can be diagnosed and the fault area of the equipment can be determined. To better process infrared images, many scholars have used image segmentation technology to conduct a lot of research and mainly divided into the traditional methods, the machine learning methods, and the deep learning methods, as shown in Table 1.

In the traditional segmentation method, Zhou et al. extract potential regions of faults by superpixel segmentation method, and then, the residual network has used to screen the real position of fault [2]. The Ostu algorithm is used to segment the image by Fan et al. To accurately segment the overheated area, the active contour model was used to refine the edge. The fuzzy C-means (FCM) clustering algorithm was used to suppress the oversegmentation, and finally, the overheated area was accurately divided [3]. In the machine learning method, Xu et al. proposed a fault region extraction method based on a pulse-coupled neural network (PCNN). This method reduces the internal parameters of the PCNN, and local features of the fault and nonfault regions are combined to achieve adaptive iteration, which can effectively extract the faulty area [5]. Shanmugam and Chandira Sekaran used the FCM clustering algorithm to segment infrared images, and the Modified Ant Lion Optimization (MALO) and Region Pros function are used to optimize the segmentation area [4]. The instance segmentation of power equipment uses the color and texture information of the equipment to segment the overall equipment, which provides a basic image for subsequent diagnosis of equipment failures. Qi et al. proposed a new method of infrared image segmentation based on a multi-information fused fuzzy clustering method. This method segmented the complete power equipment by constructing a joint domain of fuzzy clustering field (FCF) and Markov random field (MRF) [7]. Guo et al. proposed a diagnosis system based on the comprehensive analysis of infrared images. This system uses the Sobel operator and Canny operator for preprocessing, the SIFT algorithm extracts prefeature points, and the *K*-means clustering identifies power equipment [6]. With the development of deep learning, deep learning has been applied to more and more tasks. Image classification [12, 13], semantic segmentation, object detection, and instance segmentation [14, 15] have become recent academic hotspots. Infrared image segmentation based on deep learning has also been proposed by many scholars. Wang et al. used Mask R-CNN to extract the insulator instances in the infrared image, and the temperature distribution of each insulator was obtained by function fitting. This method realizes the automatic diagnosis of infrared faults of power equipment [8]. Jiang et al. used the Mask R-CNN framework to build a target detection system, which can accurately extract the bushing frame. The segmentation performance of the faulty area is improved by combining it with a pulse-coupled neural network based on linear iterative clustering [10]. Yan et al. established a multispectral instance segmentation network model based on Mask R-CNN and compared the fusion abilities of different fusion methods in detail [9]. Khalid et al. used a two-stage method of fusion-segmentation for multispectral instance segmentation. The network first uses the encoder-decoder architecture method to get the fused image and then uses Mask R-CNN for instance segmentation [11].

Although many models have been proposed based on infrared image segmentation, the current segmentation methods still need to be improved. On the one hand, most of the current segmentation methods use an infrared image dataset with distinct equipment and a clear background. When the equipment overlaps and the background is complex, these methods are challenging. On the other hand, these methods based on machine learning only use visible or infrared for segmentation, but there is a good complement of information between visible and infrared. In the deep learning method, although the visible image and the infrared image are fused by the fusion algorithm of the multispectral image, there are many redundant structures. When these algorithms are combined with the instance segmentation model, it is difficult to improve network performance. For [9], the multispectral instance segmentation based on Mask R-CNN reduces the redundant structure, but compared with the single-stage instance segmentation, the speed of the Mask R-CNN segmentation has a certain gap. This leads to practical deployment difficulties and higher costs.

To solve the above problems, this research has collected and set up power equipment image datasets, it is aimed that the complete segmentation of power equipment was realized, and a multispectral instance segmentation is designed to directly complete the classification, positioning, and pixel segmentation of power equipment. The main contributions of this work are as follows:

1. We propose a multispectral single-stage instance segmentation (MSIS) network based on SOLOv2. The method integrates image fusion and instance segmentation into a single network. The network may ensure the real-time performance of segmentation while reducing structural redundancy caused by multitasking. It may segment infrared images with complex backgrounds and poor quality, facilitating subsequent power equipment inspections.
2. To preserve more details in the original image, a dual-input feature extraction module is proposed, which can better extract the features of infrared images and visible images. It provides richer information for subsequent feature fusion and instance segmentation.
3. A multifeature attention RFN (MARFN) is proposed based on a residual fusion network (RFN), which can fuse infrared images and visible images to get a richer fusion feature. And a novel fusion layer is used to solve the problem of network degradation caused by the increase of RFN depth.

## 2. Related Works

### 2.1. Instance Segmentation

Instance segmentation is an instance-level object segmentation method in image segmentation tasks. Instance segmentation is mainly divided into two stages and a single stage, as shown in Table 2. The popular instance segmentation [14, 16–19] is to find out the area where the instance is located through the method of object detection, and then, semantic segmentation is performed in the detection box. Each segmentation result is output as a different instance. In methods such as SGN [20] and SSAP [21], pixel-level semantic segmentation is first performed, and then, different instances are distinguished by means such as clustering and metric learning. Most single-stage instance segmentation methods [15, 22–24] are mainly inspired by one-stage and anchor-based detection models such as YOLO [27] and RetinaNet [28]. PolarMask [25] and AdaptIS [26] are inspired by anchor-free detection models such as FCOS [29]. Compared with the two-stage model, the single-stage model has a natural advantage in speed [15].

### 2.2. Image Fusion

There are four categories of image fusion algorithms based on deep learning, mainly including the CNN method, the GAN method, the self-encoding method, and other methods, as shown in Table 3.

The image fusion method based on CNN mainly uses the existing CNN network for image fusion. Li et al. proposed an image fusion network based on VGG-19 [32], which decomposes the source image into two parts: the basic part and the detailed content, then the VGG-19 is used to extract multilayer features, and the fusion image is obtained through an appropriate fusion strategy. Li et al. used residual neural network (ResNet) and zero-phase component analysis (ZCA) to construct a fusion framework. The residual neural network was used for feature extraction, and the image was reconstructed by zero-phase component analysis [33]. Inspired by the transform-domain image fusion algorithms, Zhang et al. used two convolutional layers to extract the salient image features of multiple images, and appropriate fusion rules were selected to fuse these features and generate images [31]. The shortcomings of the network are also obvious. The structure and fusion strategy are too simple, so the fusion performance of the network is not optimal. In the paper [30], an unsupervised and unified densely connected network (FusionDN) is proposed. It is the main contribution that the weights of different source images were generated by weight block, which is to complete the fusion of different source images. Zhang et al. proposed a fast unified image fusion network based on proportional maintenance of gradient and intensity (PMGI), which can fuse multisource images [35]. The fusion result is achieved by adjusting the texture and intensity ratio of the image. In the network, the information is extracted through the gradient path and the intensity path. In order to meet the fusion task of different sources, the author also defines two loss functions for extracted information. Xu et al. provide a fusion network model that adapts to different source images because the model can retain the adaptive similarity between the fusion result and source images [36]. Chen et al. designed a multilayer fused convolution neural network (MLF-CNN) for pedestrian detection; they combined image fusion and object detection into a single network [34].

The autoencoder method uses the existing autoencoder neural network to extract features, fuse features, and generate features. Prabhakar et al. proposed a fusion network from the perspective of optimizing the loss function. The network is composed of an encoder, a fusion layer, and a decoder [37]. Even if the network input changes and the parameters are not adjusted, better results can be obtained. Inspired by DeepFuse, a fusion network based on an autoencoder neural network [38] was proposed by Li and Wu. The network is composed of an encoder, a fusion layer, and a decoder. The dense block [45] is mainly used for feature extraction of the original image. NestFuse [39] also uses the same structure, which is inspired by DenseFuse and U-Net++ [46]. The author also designed a multiscale fusion strategy based on the attention mechanism. In 2021, Li et al. proposed an end-to-end residual fusion architecture (RFN-Nest). Its main contribution was to design a residual fusion network (RFN) based on the residual architecture [40].

In the GAN-based approach, the Generative Adversarial Network is used to train a generator that can generate fused images. An image fusion framework based on generative adversarial networks [41] was proposed by Ma et al. The generator is used to generate the fusion image, and the discriminator is used to discriminate the result of the generator. But the network still cannot retain the rich detail. To preserve the rich details in the visible image, the author improves FusionGAN [42]. The author has improved the generator, discriminator, and loss function of the GAN network. These changes make the fused image have more details. As a network that solves the fusion task, there are problems such as poor real-time performance of the network due to structural redundancy when it is combined with the instance segmentation for multiple networks.

Other methods are different from the above methods. In the paper [43], the input infrared image and visible image are decomposed into three high-frequency feature images and low-frequency feature images, then, a specific fusion strategy is used to fuse two sets of feature images, and the fusion image is obtained through image reconstruction. The paper [44] proposed an infrared and visible image fusion method based on multiscale transformation and norm optimization. The fusion ability of the network as a whole was improved by using a combination of prefusion and postfusion in the paper.

Image fusion methods based on CNN, GAN, and other types are independent structures, which makes it relatively difficult to combine with instance segmentation networks and also produces structural redundancy. The self-encoding method can be combined with the existing instance segmentation method in a modular form to avoid the above-mentioned problems. Therefore, this paper builds our multispectral feature fusion module based on the RFN of the RFN-Nest method.

## 3. Materials and Methods

### 3.1. MSIS Network Architecture

The architecture of the MSIS model is shown in Figure 1, which consists of three parts: feature extraction module, feature fusion module, and the module of multiscale instance segmentation. Firstly, the feature extraction module generates infrared image features {FM_*ir*,*i*_}_*i*=1_^4^, visible image features {FM_*vi*,*i*_}_*i*=1_^4^, and prefusion features {FM_*pf*,*i*_}_*i*=1_^4^ from the input infrared image *I*_*ir*_ and visible image *I*_*vi*_. Then, in order to obtain the fused features {FM_*mi*_}_*i*=1_^4^, these features are input to the feature fusion module (MARFN).

In the module of multiscale instance segmentation, FPN (Feature Pyramid Network) was used by MSIS to improve the ability of multispectral instance segmentation and deal with the multiscale problems of power equipment in SOLOv2. The FPN can fuse deep semantic features and shallow detail features. These new features were input into the prediction head of the multispectral instance for prediction. Here, we use the prediction header of SOLOv2, including the instance category branch and instance mask branch. The specific operation is as follows: the feature of FPN output will be divided into *S* × *S* grids. The branch of the instance category will output *S* × *S* × *C* semantic category probabilities, where *C* is the number of instance categories. The branch of instance mask outputs *H* × *W* × *S*^2^ prediction masks, *H* × *W* represents the size of the output image, and *S*^2^ is the maximum number of instances predicted. When the center position of the target object falls into a certain grid, its corresponding category branch and mask branch will output the object instance category and pixel segmentation, respectively. Finally, MSIS realized the end-to-end feature fusion and automatic segmentation of complete power equipment.

### 3.2. MSIS Feature Extraction Module

Before the feature fusion of infrared image *I*_*ir*_ and the visible image *I*_*vi*_, feature extraction is an indispensable step. However, the difficulty in the training of the network model is due to the limited amount of data in the power equipment dataset. And the pretrained ResNet-50 model on the MS COCO dataset was used for feature extraction; the segmentation effect is not very satisfactory. To this end, we propose the MSIS feature extraction module, including the feature extraction branch of the infrared image, the feature extraction branch of the visible image, and the feature prefusion branch. Specifically, as shown in Figure 2, the feature extraction branch of the visible image and the feature extraction branch of the infrared image use the pretrained ResNet-50. The feature prefusion branch is composed of 2 3 × 3 Conv, attention mechanism, and residual structure (Stage 1–Stage 3). In the structure, 3 × 3 Conv is to ensure that the input feature information is fully retained, and the number of output channels is 512. We add 1 × 1 Conv before each residual structure, ensuring that the output is consistent with ResNet-50 features. And at the same time, it can effectively reduce the computational burden, which was caused by the increase of channels because the training parameters were reduced by dimensionality reduction. The residual structure is consistent with the structure in ResNet-50. Meanwhile, the attention module is added behind each residual structure. The channel attention module (CA) and the spatial attention module (SA) are a parallel combination. The feature FM_*am*_ generated by its attention module can be equivalent to the expression (1).

(1) $$\begin{array}{c} {\text{FM}}_{am}^{\prime }=\text{SA}\left({\text{FM}}_{pf}\right)+\text{CA}\left({\text{FM}}_{pf}\right). \end{array}$$

### 3.3. MSIS Feature Fusion Module

The feature fusion module of the MSIS is responsible for the task of fusing infrared image features {FM_*ir*,*i*_}_*i*=1_^4^ and visible image features {FM_*vi*,*i*_}_*i*=1_^4^. The MSIS feature fusion module is based on the RFN module, as shown in Figure 3. In the original RFN structure, the convolution size is 3 × 3 Conv.

The original intention of RFN's fusion layer fusion convolutional layer (Conv3∼Conv6) is to fuse features from different sources through the convolutional layer, but the convolutional fusion ability of the fusion layer is not very good; see ablation experiment of fusion layer for details. We try to increase the number of convolutional layers and modify the convolutional layer to improve the fusion ability of the fusion layer. In the case of enhancing the ability of feature fusion and ensuring fewer module parameters, we construct a novel multifeature attention RFN (MARFN), as shown in Figure 4. The features of the infrared image FM_*ir*_ and the features of the visible image FM_*vi*_ are spliced by channels through Conv1 and Conv2, and Space Attention is arranged after Conv1 and Conv2.

Then, they are input into the fusion convolutional layer (Conv3∼Conv6). The increase in the number of convolutional layers will cause degradation. In order to solve this problem, we design a new convolutional layer. As shown in Figure 5, this structure can well solve the phenomenon of degradation caused by the increase in the number of layers in the module.

Finally, the prefusion features FM_*pf*_ in the MARFN-A will be input into Conv7, and Conv7 will combine the output of Conv3∼Conv6 into the next layer and get the fusion feature FM_*m*_. After Conv3∼Conv7, the channel attention (CA) will be placed. According to Figure 4(a), the feature fusion formula is defined as shown in

(2) $$\begin{array}{c} {\text{FM}}_{m}=F\left({\text{FM}}_{vi},{\text{FM}}_{ir},{\text{FM}}_{pf}\right). \end{array}$$

The MARFN-B is different from the MARFN-A; FM_*vi*_ and FM_*ir*_ will be input into Conv7 at the same time. According to Figure 4(b), the feature fusion formula is defined as shown in

(3) $$\begin{array}{c} {\text{FM}}_{m}=F\left({\text{FM}}_{vi},{\text{FM}}_{ir}\right). \end{array}$$

### 3.4. Loss Function

In order to accelerate the convergence of the fusion module, we have added a new branch to calculate the loss of feature fusion. The loss is defined as follows:

(4) $$\begin{array}{c} L_{\text{fusion}}=\sum w_{l}\left(w_{vi}{\left\|{\text{FM}}_{m}-{\text{FM}}_{vi}\right\|}_{F}^{2}+w_{ir}{\left\|{\text{FM}}_{m}-{\text{FM}}_{ir}\right\|}_{F}^{2}\right). \end{array}$$

*w*_*l*_ is the loss coefficient of different feature layers, and *w*_*vi*_ and *w*_*ir*_ are used to balance the loss of each scale in the multiscale features. FM_*vi*_ and FM_*ir*_ control the relative influence of visible and infrared features in the fusion feature map FM_*m*_. The MARFN fuses the features of the infrared image FM_*ir*_ and the visible image FM_*vi*_ to generate the features FM_*m*_ required by the FPN. The multiscale instance segmentation module can obtain the final instance segmentation results. We use the SOLOV2 single-stage prediction head, so the loss definition of the multiscale instance segmentation module is consistent with SOLOv2, and its definition is as follows:

(5) $$\begin{array}{c} L=L_{\text{cate}}+L_{\text{mask}}. \end{array}$$

*L*_cate_ means focal loss, *L*_mask_ means dice loss, and more details about loss function can be found in SOLOV2. Therefore, our total loss is defined as follows:

(6) $$\begin{array}{c} L=\alpha L_{\text{cate}}+\beta L_{\text{mask}}+\gamma L_{\text{fusion}}. \end{array}$$

## 4. Results and Discussion

### 4.1. Image Dataset of Power Equipment

The image dataset of power equipment comes from a medium-sized converter station in Huanggang City, Hubei Province, China. In the experiment, we constructed and used this dataset, and all infrared images and visible images were obtained by an infrared thermal camera (Fluke Ti480 PRO). The shooting time is from 8 : 00 am to 5 : 00 pm, and the weather is mainly cloudy and sunny. The image mainly contains common power equipment such as transformers and lightning arresters. The power equipment dataset is shown in Figure 6. The power equipment dataset is mainly used for image processing tasks such as object detection and instance segmentation. In the experiment of the multispectral instance segmentation, we used the method [47] to obtain the final registration image. The multispectral image consists of 2940 pairs of arresters and 2998 pairs of transformers. The division ratio of the training set, validation set, and test set is 6 : 2 : 2, and the distribution results of the power equipment dataset during training are shown in Table 4. The dataset is manually labeled by LabelMe. And according to the MS COCO dataset style, we constructed a dataset of instance segmentation.

### 4.2. Experiment Setup

The experiment was completed on a deep learning server, which was configured with NVIDIA Tesla V100 GPU and Intel(R) Xeon(R) CPU E5-2673 v3 @ 2.40 GHz, the OS was 64-bit Ubuntu 18.04, and the network was implemented based on Pytorch 1.3.0. In model training, it is *L*_fusion_ that the loss function is used by the multispectral fusion network, and *L*_cate_ and *L*_mask_ are used by the loss functions of the multispectral instance segmentation network. We use stochastic gradient descent (SGD) as the optimizer during network training, and its learning rate (lr) is 0.01, the momentum parameter (momentum) is 0.9, and the decay value (decay) of the learning rate for each update is 0.0001. The evaluation index is the detection evaluation index of COCO [48], including AP, AP^50^, AP^75^, AP^*S*^, AP^*M*^, and AP^*L*^.

### 4.3. Our Results

To validate the proposed MSIS model, we quantitatively and qualitatively evaluate the MSIS model with existing state-of-the-art methods on multispectral datasets of electrical devices, which include two-stage, single-stage, and multispectral instance segmentation. The two-stage instance segmentation contains Mask R-CNN [14], MS R-CNN [17], TensorMask [18], and PANet [16]. The single-stage instance segmentation has PolarMask [25], YOLACT++ [24], and SOLOv2 [15], and multispectral has Mask R-CNN (RFN) [11], SOLOv2 (RFN), and Mask R-CNN (^*∗*^) [43]. In the above instance segmentation network, the two-stage and single-stage instance segmentation methods only use infrared light images. Multispectral instance segmentation includes instance segmentation based on image fusion (Mask R-CNN (RFN) and SOLOv2 (RFN)) and instance segmentation based on feature fusion (Mask R-CNN (^*∗*^) and MSIS). In instance segmentation based on image fusion, the RFN-Nest method is used for image fusion, and then, the fused image will be input to the instance segmentation. In instance segmentation based on feature fusion, different fusion strategies are used to fuse features, and then, instance segmentation is performed based on the fusion features. The quantitative evaluation results of the above network are shown in Table 5.

In Table 5, the AP value of the MSIS model based on ResNet-101 reaches 42.20%, which is better than the other methods above to achieve the segmentation of power equipment. Compared with SOLOv2, which only uses infrared images, the effect is significantly improved, and the AP value is increased by 7.5%. The reason is that MSIS can obtain information of infrared images and visible light images at the same time, and the complementarity of information improves the semantic information processing capabilities of the network. Compared with SOLOv2 (RFN), the AP value of MSIS has increased by 3.4%. This shows that the proposed prefusion network and MARFN module can obtain richer fusion features than the RFN module. We also evaluated the FPS of MSIS on the NVIDIA Tesla V100 GPU, as shown in Table 6. The MSIS based on Res-50-PFN can reach 12 FPS, and the lightweight model based on SOLOv2 can reach 23 FPS.

For further explanation, Figure 7 shows the segmentation results of the above method on the power equipment multispectral dataset. (c) and (d) represent instance segmentation using only infrared light images, and they show the phenomenon of incorrect segmentation of overlapping objects. The reason is that the lower resolution results in no clear boundary between overlapping objects. (e) and (f) represent the result of segmentation RFN fusion. Although the problem of incorrect segmentation in (c) and (d) is solved, the accuracy of object boundary segmentation is not very high because the fusion capability of the RFN module is poor. At the same time, the large network and redundant structure make it difficult to improve network speed. (g) and (h) are the fusion of the feature-level, which reduces the redundancy of the network structure and improves the performance at the same time. The MSIS model fuses the feature of the infrared image and the feature of the visible image, which makes the object boundary more accurate. Compared with the Mask R-CNN (^*∗*^), the single-stage model based on SOLOv2 has certain advantages in speed. The segmentation results show that the segmentation accuracy of the MSIS model is improved under complex backgrounds, multiple targets, and changes in illumination circumstances.

This article provides generalization experiments to prove the effectiveness of the proposed method. The MSIS method is tested on the FLIR thermal imaging dataset. The FLIR thermal imaging dataset was provided by FLIR for ADAS and driverless technology, which mainly includes thermal images and RGB images. Since the FLIR thermal imaging dataset provides annotation information for target detection, the object detection prediction head will be used to complete the generalization experiment. In Table 7, Faster R-CNN represents the original network. Faster R-CNN (MSIS) uses the proposed MISS method and replaces the prediction head with the prediction head of Faster R-CNN. As shown in Table 7, the mAP of Faster R-CNN (MSIS) is 58.56, which is 5.22% higher than Faster R-CNN. This result is basically consistent with the result of the MS COCO dataset.

### 4.4. Ablation Experiment

In this section, in order to verify the superiority of the proposed MSIS method, we provide four sets of ablation experiments. They are the ablation experiment of the feature fusion module, the ablation experiment of the fusion layer, the ablation experiment of the backbone, and the ablation experiment of the prefusion network. The experimental process is as follows. First, the ablation experiment of the fusion layer and the ablation experiment of the feature fusion module are executed. Next, the best fusion layer and feature fusion module are used for ablation verification of the prefusion network. When the above-mentioned ablation experiment is completed, the main ablation experiment is finally carried out.

#### 4.4.1. Ablation Experiment of Fusion Layer

In the fusion layer ablation experiment, we consider the fusion convolutional layer from two perspectives: the number of convolutional layers and the structure of the convolutional layer. RFN (Conv × 3) represents the original fusion convolution layer, which means that only 3 layers of convolution are provided. RFN (Conv × 4) to RFN (Conv × 6) indicate that 4, 5, and 6 layers of convolution are provided, respectively. Fusion Convolutional Layer (Conv × 6) represents the proposed fusion layer convolution. The comparison results are shown in Table 8.

In Table 8, after the fusion convolutional layer is increased to 5 layers, the fusion ability of the network decreases. This also causes the AP value to drop further. The main reason is that the network is degraded. In the process of forward transmission, as the number of convolutional layers increases, the image information contained in the feature map will decrease layer by layer. The deep network may get a worse training effect than the shallow network. Based on this analysis, we propose a new fusion layer structure, as shown in Figure 7. In Table 8, we compare the performance brought by different fusion layers. When the number of FCL increases to 6, the network segmentation ability still maintains good fusion performance.

#### 4.4.2. Ablation Experiment of Feature Fusion Module

This section compares the MSIS feature fusion module with the existing fusion methods (Add, Max, *l*_1_ − norm, *l*_*∗*_ − norm, SCA and RFN). In the existing fusion module, add refers to directly adding different features. Max selects the maximum value of the element as the fusion feature. The method based on *l*_1_ − norm refers to calculating the weight based on *l*_1_ − norm. The *l*_*∗*_ − norm (known as nuclear-norm) method refers to obtaining the fusion weight by calculating the sum of singular values of a matrix involved in the global pooling operation of deep features. SCA represents the spatial/channel attention fusion strategy used in NestFuse [39]. RFN represents the residual fusion strategy used in RFN-Nest. The expression definition is shown in Table 9.

We use 6 evaluation indicators for evaluation. They include Entropy (En) [49], Standard Deviation (SD) [50], Mutual Information (MI) [51], Improved Fusion Artifact Measurement (*N*_*abf*_) [52], Sum of Difference Correlation (SCD) [53], and Multiscale Structural Similarity (MS-SSIM) [54]. At the same time, in order to evaluate the indicators, Nest-RFN will be used as the basic fusion network. The different fusion images are obtained by replacing the strategy fusion of the Nest-RFN. Finally, the fusion result quality index evaluation table is shown in Table 10.

In Table 10, the fusion methods based on convolution (SCA, RFN, MARFN-A, and MARFN-B) get better fusion effects than other classic fusion methods. From the perspective of information retention (En, SD), the fusion methods based on convolution extract rich image features through convolution, and these features are used by the fusion convolution structure to generate fused features. Finally, a better result than the classic fusion method is obtained. Although both MARFN-B and RFN are fusion methods based on convolution, the MARFN-B method is better than RFN. The main reason is that FCL can further improve the fusion of features and retain richer information. In addition, MARFN-A has a significant improvement in the evaluation indicators. From the perspective of feature preservation (MS-SSIM, MI), the prefusion network and MARFN-A construct deeper feature extraction and fusion, thereby enhancing the fusion capability.

#### 4.4.3. Ablation Experiment of Prefusion Network

In the ablation experiment of the prefusion network, two sets of experiments are provided; they are MARFN-B, and MARFN-A based on the prefusion network. The experimental results are shown in Table 11. “✓” means that the prefusion network is enabled. The MARFN-A module with a prefusion network has been significantly improved, and its AP value has increased by 5%. The prefusion network provides richer features and enhances the fusion capability of the MARFN module, and finally, the overall segmentation performance of the network is improved.

#### 4.4.4. Ablation Experiment of Backbone

To explore the feature extraction module in the MSIS, in the ablation experiment of the MSIS backbone, we provide two backbones. They are dual-input backbone based on the traditional backbone and dual-input backbone based on the feature extraction module of the MSIS, respectively. Dual-input backbone based on traditional backbone uses the classic backbone (ResNet-101 or ResNeXt-101), whose structure is shown in Figure 8. Dual-input backbone based on the feature extraction module of the MSIS is a combination of the MSIS feature extraction network and the classic backbone (MSSIS_ResNet−101_ or MSSIS_ResNeXt−101_), as shown in Figure 2.

Table 12 shows the performance of network segmentation for different backbones. Compared with ResNet-101, the AP value has increased by 4.54%. The AP of the MSSIS_ResNeXt−101_ reached 43.61%. From the perspective of feature extraction, the backbone based on the feature extraction module of the MSIS provides rich features for the MARFN module. They include not only infrared light image features and visible light image features but also prefusion features. From the perspective of feature fusion, the combination of prefusion network and MARFN extracts more complex features and provides deeper feature fusion, thereby enhancing the fusion capability of the fusion network.

## 5. Conclusions

In this work, we designed an end-to-end multispectral instance segmentation model, which can achieve complete segmentation of power equipment and meet the requirements of the preliminary work of power fault detection and segmentation for nonfaulty equipment. Compared with ordinary instance segmentation, the proposed network adds a multispectral feature fusion network to fuse the features of infrared images and visible images. For the MSIS network model, we have done enough experiments and adopted the best solution to greatly improve the accuracy of segmentation. To better process infrared images and visible images, we propose a dual-input method, which takes advantage of the advantages of infrared images and visible light images at the same time. Finally, the AP of the MSIS model reached 40.06%, and the segmentation results can be seen in Figure 7. The multispectral instance segmentation can achieve complete segmentation of power equipment and help with power equipment fault detection, however, there is no segmentation of faults, and the model itself belongs to a large model to be further optimized. Therefore, in future research, the model will be further improved for fault detection.

## Figures and Tables

**Figure 1:** MSIS model architecture. (a) MSIS feature extraction module. (b) MSIS feature fusion module. (c) MSIS multiscale instance segmentation module.

**Figure 2:** The feature extraction module. (a) The feature extraction branch of the infrared image. (b) The feature extraction branch of the visible image. (c) The prefused feature extraction branch. The feature extraction branch of prefusion is composed of 3 × 3 Conv, 1 × 1 Conv, residual structure (Stage 1–Stage 3), spatial attention (SA), and channel attention (CA).

**Figure 3:** The architecture of RFN. Conv1∼Conv5 represents convolutional layers.

**Figure 4:** The architecture of MARFN, (a) represents MARFN-A, (b) represents MARFN-B, Conv1∼Conv3 represents convolutional layers, SA and CA represent spatial attention and channel attention modules, respectively, and FCL1∼FCL4 represent fusion convolutional layer.

**Figure 5:** Fusion convolutional layer (FCL). FM_*n*−1_ represents the output feature of the previous layer, and FM_*n*_ represents the output feature of this layer.

**Figure 6:** Power equipment dataset.

**Figure 7:** The segmentation results of different methods in the power equipment dataset, where (a) represents the visible light image, (b) represents the infrared light image, (c) represents segmentation results of the MS R-CNN method, (d) represents segmentation results of SOLOv2 method, (e) represents segmentation results of Mask R-CNN(RFN) method, (f) represents segmentation results of SOLOv2(RFN) method, (g) represents segmentation results of Mask R-CNN(^*∗*^) method, and (h) indicates segmentation results of MSIS method.

**Figure 8:** Structure diagram of multispectral feature extraction based on the traditional backbone.

**Table 1:** The segmentation method of infrared image.

Category	Method	Advantage	Disadvantage
The traditional method	[2, 3]	(i) Fast running	(i) Sensitivity to noise
		(ii) Low hardware requirements	(ii) Excessive segmentation

The machine learning methods	[4–7]	(i) Logical interpretability	(i) Complex feature engineering
		(ii) Low hardware requirements	

The deep learning methods	[8–11]	(i) Strong learning ability	(i) Large number of training samples
		(ii) Good generalization ability	(ii) Higher hardware requirements

**Table 2:** Instance segmentation method.

Category	Method	Advantage	Disadvantage
Two stage	[14, 16–21]	(i) High precision	(i) Low speed
Single stage	[15, 22–26]	(i) High speed	(i) Low precision

**Table 3:** Segmentation method of infrared image.

Category	Method	Advantage	Disadvantage
The CNN method	[30–36]	(i) Richer features	(i) Poor fusion ability
The self-encoding method	[37–40]	(i) End-to-end approach (ii) Modular structure	(i) Complex loss function design
The GAN method	[41, 42]	(i) Special method	(i) Difficulty in optimization
Other methods	[43, 44]	(i) Higher accuracy	(i) Poor commonality

**Table 4:** The distribution result of the power equipment dataset during training.

Class name	Training set	Validation set	Test set	Total
MOA	1764	588	588	2940
CT	1800	599	599	2998

**Table 5:** The quantitative evaluation results of the above network.

Method	Backbone	AP	AP^50^	AP^75^	AP^*S*^	AP^*M*^	AP^*L*^
Mask R-CNN	Res-101-FPN	32.67	51.63	34.76	—	10.45	33.52
MS R-CNN	Res-101-FPN	35.21	55.76	38.43	—	11.55	32.51
TensorMask	Res-101-FPN	34.04	56.26	36.36	—	11.26	29.76
PANet	Res-50-FPN	33.54	54.93	36.21	—	11.26	31.23
PolarMask	Res-101-FPN	27.34	48.84	27.94	—	10.54	30.96
YPLACT++	Res-101-FPN	31.53	50.74	33.84	—	14.90	33.23
SOLOv2	Res-101-FPN	34.63	52.66	35.84	—	11.01	46.57
Mask R-CNN (RFN)	Res-101-FPN	37.81	61.51	38.54	—	13.20	39.41
SOLOv2 (RFN)	Res-101-FPN	38.77	62.77	42.14	—	16.44	49.52
Mask R-CNN (^*∗*^)	Res-101-FPN	37.97	61.46	39.05	—	15.20	52.70
MSIS	Res-50-FPN	40.06	63.26	45.62	—	17.61	62.37

**Table 6:** The FPS results of MSIS.

Model	FPS
MSIS (Res-50-PFN)	12
MSIS (lightweight)	23

**Table 7:** The MSIS results on FLIR thermal dataset.

Model	mAP
Faster R-CNN	58.56
Faster R-CNN(MSIS)	63.34

**Table 8:** The results of experiments with different fusion layers.

Fusion layer	AP	AP^50^	AP^75^
RFN (Conv × 3)	37.16	60.37	42.78
RFN (Conv × 4)	38.21	61.39	43.74
RFN (Conv × 5)	36.23	59.42	41.73
RFN (Conv × 6)	35.20	58.39	40.74
FCL (Conv ×6 )	40.22	63.37	45.72

**Table 9:** Ablation experiment of feature extraction module in MSIS network.

Fusion module	Expression
Add	FM_*f*_=FM_*ir*_+FM_*vi*_
Max	FM_*f*_=max(FM_*ir*_, FM_*vi*_)
*l*_1_ − norm	FM_*f*_=*l*_1_(FM_*ir*_, FM_*vi*_)
*l*_*∗*_ − norm	FM_*f*_=*l*_*∗*_(FM_*ir*_, FM_*vi*_)
SCA	FM_*f*_=SCA(FM_*ir*_, FM_*vi*_)
RFN	FM_*f*_=RFN(FM_*ir*_, FM_*vi*_)
MARFN-A	FM_*m*_=MARFN − *A*(FM_*ir*_, FM_*vi*_, FM_*pf*_)
MARFN-B	FM_*m*_=MARFN − *B*(FM_*ir*_, FM_*vi*_)

**Table 10:** Ablation experiment of MSIS feature fusion module.

Fusion module	En	SD	MI	*N*_*abf*_	SCD	MS-SSIM
Add	6.799	67.56	13.5	0.204	1.965	1.062
Max	6.834	92.621	13.565	0.332	1.707	0.915
*l*_1_ − norm	6.953	93.336	13.774	0.339	1.691	0.874
*l*_*∗*_ − norm	6.918	73.799	13.753	0.209	1.911	1.038
SCA	7.027	82.877	13.948	0.25	1.853	0.989
RFN	6.978	72.031	13.821	0.21	1.976	1.028
MARFN-A	7.182	74.154	14.142	0.342	2.195	1.345
MARFN-B	7.055	74.014	14.008	0.201	2.057	1.242

**Table 11:** The refusion network ablation experiment results.

Prefusion network	AP	AP^50^	AP^75^
✓	35.38	58.53	40.85
	40.38	63.49	45.84

**Table 12:** Ablation experiment results of feature extraction modules of different backbones.

Backbone	AP	AP^50^	AP^75^
ResNet-101	38.87	62.90	42.29
ResNeXt-101	40.13	64.84	43.57
MSSIS_ResNet−101_	42.33	66.55	46.96
MSSIS_ResNeXt−101_	43.61	68.64	48.36

## Data Availability

The data used to support the findings of this study are available from the corresponding author upon request.
